RETRACTED

# Effect of Peptidylarginine Deiminase 4 on Endothelial Progenitor Cell Function in Peripheral Arterial Disease

**DOI:** 10.1155/2021/7550693

**Published:** 2021-07-26

**Authors:** Jialin Pan, Wenqin Liu, Ye Chen, Chi Zhang, Cong Lin

**Affiliations:** Department of Cardiology, The Second Affiliated Hospital of Wenzhou Medical University, Wenzhou 325000, Zhejiang, China

## Abstract

At present, the global prevalence of peripheral arterial disease is increasing year by year, and it has become a worldwide disease. Studies have shown that transplanting endothelial progenitor cells (EPCs) into ischemic tissues can improve the tissue ischemia, thereby having a therapeutic effect on peripheral arterial diseases. This indicates that EPCs play a therapeutic effect in peripheral arterial disease. Recent studies have shown that peptidylarginine deiminase (PAD) is involved in the regulation of epigenetics and its inhibitor Cl-amidine can improve endothelium-dependent vasodilation and significantly reduce the formation of arterial thrombosis. It can also play a role in hematopoietic stem cells that share the same origin with EPCs. Therefore, we speculate that PAD4 may also have an effect on EPCs through a similar mechanism, thereby participating in the damage and repair of peripheral arterial disease. Therefore, we first detected the expression of PAD4 in EPCs of peripheral arterial disease and detected changes in the number and function of endothelial progenitor cells in peripheral blood after injecting the PAD4 inhibitor Cl-amidine into mice. A mouse model of lower limb ischemia was established to explore the effect of PAD4 on the function of EPCs in peripheral arterial disease. The results show that PAD4 is highly expressed in peripheral arterial diseases and the PAD4 inhibitor Cl-amidine can increase the number of EPCs and can treat peripheral arterial diseases by improving the proliferation, migration, and vascularization of EPCs.

## 1. Introduction

Peripheral artery disease (peripheral artery disease) is a common circulatory system disease caused by limb ischemia caused by arterial vascular stenosis. Its main clinical manifestation is systemic diffuse atherosclerosis. According to statistics, the current global prevalence of peripheral artery disease is about 3–12% [1]. Among them, low- and middle-income countries are the hardest hit areas for peripheral arterial disease (approximately 70% of the number of patients), and peripheral arterial disease has become a major worldwide disease. Fowkes et al. [2] reported in 2010 that about 200 million people in the world were currently affected by peripheral arterial disease to varying degrees. As an important disease currently attracting attention, it is necessary to conduct active research on the pathogenic mechanism of peripheral vascular disease and corresponding treatment measures. Although surgical treatments and medical treatments have been proposed, the existence of surgical risks and drug side effects makes it necessary to explore safer and effective treatment methods to avoid the shortcomings of current treatments.

RETRACTED

Studies have shown that direct transplantation of endothelial progenitor cells (EPCs) into ischemic tissue can improve tissue ischemia, thereby achieving the therapeutic effect of peripheral arterial disease [3]. However, under normal circumstances, the number of EPCs circulating in the peripheral blood is quite low (the number in white blood cells is only about 0.02%–0.06%), and the limit of the number makes it insufficient to effectively exert the repair effect on ischemic tissue [4]. Therefore, how to make more endothelial progenitor cells appear in the peripheral blood of the body so that more endothelial progenitor cells can enter the ischemic tissue to achieve the effect of speeding up the treatment is a problem that we urgently need to think about and solve.

Recent studies have shown that peptidylarginine deiminase (PAD) is involved in the regulation of epigenetics. As a calcium-dependent protease, it is distributed in the epidermis, skeletal muscle, and brain. In many tissues and organs of the body, it has the function of converting arginine residues bound to polypeptides into citrulline [5]. Darrah et al. [6] found that PAD4 can participate in the pathological process of rheumatoid arthritis through the inhibition of antithrombin. Slack et al. [7] found that the peptide acyl arginine deiminase 4 inhibitors F-amidine and Cl-amidine have killing effects on a variety of tumor cell lines. In addition, the study of Nakashima et al. [8] confirmed that PAD4 can affect the proliferation of pluripotent hematopoietic stem cells by regulating the expression of C-myc gene. From the perspective of cell origin, hematopoietic stem cells and endothelial progenitor cells are derived from a common precursor cell, and their biological behaviors are similar [9]. We speculate that PAD4 may be involved in the repair of vascular disease damage through a similar mechanism. Plerixafor (AMD3100) is a CXC chemokine receptor 4 (CXCR4) antagonist, which can mobilize endothelial progenitor cells and circulating angiogenesis to treat lower limb ischemia. Therefore, this experiment uses AMD3100 as the positive control for this study. We first detected the presence of PAD4 expression in EPCs, and detected changes in the number and function of endothelial progenitor cells in peripheral blood by injecting the PAD4 inhibitor Cl-amidine into mice. A mouse model of lower limb ischemia was established to explore the effect of PAD4 on the function of EPCs in peripheral arterial disease. The specific report is as follows.

RETRACTED

## 2. Materials and Methods

### 2.1. Cell Source and Culture

The peripheral blood of healthy volunteers and patients with peripheral arterial disease was collected, placed in a test tube of 2500 IU heparin, and immediately transferred to the laboratory. All volunteers signed an informed consent form voluntarily. The EPCs were separated immediately, and the peripheral blood was diluted 1 : 1 and placed in a centrifuge tube. The diluent and the lymphocyte separation liquid were separated (the upper and lower liquid volume ratio was 2 : 1), and a clear interface was visible. The liquid in the centrifuge tube was divided into 4 layers after centrifugation at 2000 r/min and 20 min. From top to bottom, there was a diluent layer, a mononuclear cell layer (a ring-shaped milky white layer), a transparent separating liquid layer, and a red blood cell layer. The mononuclear cell layer was aspirated and added to a centrifuge tube (added 5 times the volume of PBS), mixed well, centrifuged at 1500 r/min for 15 min and washed twice, and then centrifuged; then the supernatant was discarded and EGM-2 complete medium was added to resuspend cell. Then we counted, adjusted the cell density to 1 × 10^6^/mL, inoculated it in a culture flask precoated with FN, and cultured it in a constant temperature incubator at 37°C and 5% CO_2_. We changed the medium for the first time after 8 hours, observed and recorded the cell growth morphology, and changed the medium every 3 days. After cultivating for 10 days, the cells in good growth state were subcultured, and the cell density was adjusted to 1 × 10^6^/mL and seeded in various well plates or Petri dishes for subculture. Dil-labeled low-density lipoprotein (Dil-LDL) was used for the identification of EPCs.

### 2.2. RNA Extraction and Real-Time Quantitative PCR Determination

The Qiagen RNeasy Mini kit was combined with on-column DNA enzyme treatment (Applied Biosystems, Foster City, CA, USA) to isolate total RNA from cells. High-capacity RNA-to-cDNA kit (Applied Biosystems) was used to synthesize the first strand of cDNA. QRT-PCR was performed using Power SYBR Green PCR Master Mix (Applied Biosystems) and gene-specific primers. The primer sequence PAD4:5-TGTCCGTCAGAACCCATGC-3(F):5-CATGTTCCACCACTTGAAGG-3(R), GAPDH:5-ACCCATCACCATCTTCCAGGAG-3(F); 5-ACCCATCACCATCTTCCAGGAG-3(F). 2^−ΔΔCt^ was used to calculate the relative expression of the detected gene. △△CT(n) = △Ct(n) − △Ct(1); △Ct(n) = Ct target gene (n)-Ct internal reference gene (n).

RETRACTED

### 2.3. Localization of PAD4 in Cells

The cells were grown on glass slides in 12-well plates, then fixed with 4% paraformaldehyde, and permeabilized with 0.1% Triton X-100. After blocking, the cells were incubated with primary antibodies against Flag and GSK3*β*. Then Fluor 555 combined with goat anti-mouse secondary antibody (Invitrogen, Carlsbad, CA, USA) or Fluor 488 combined with goat anti-rabbit secondary antibody (Invitrogen) was used to detect fluorescence. The nuclei were stained with DAPI (Vector Laboratory, Cambridgeshire, UK). A representative image was collected using a Carl Zeiss LSM 510 laser scanning confocal microscope.

### 2.4. Animal Source

60 male C57BL/6N mice (Beijing Weitong Lihua Experimental Animal Technology Co., Ltd.) were adaptively fed for 1 week, and 30 of them were divided into three groups: (1) PBS group (subcutaneous injection of PBS 10 mg/kg)), (2) Cl-amidine group (subcutaneous injection of Cl-amidine 10 mg/kg), and (3) AMD3100 group (subcutaneous injection of AMD3100 5 mg/kg in the abdomen). All mice were maintained in a specific pathogen-free environment. After 14 weeks, the peripheral blood of the mice was collected, and the mononuclear cells were isolated and stored. All animal experiments were approved by the Animal Experiment Ethics Committee of Wenzhou Medical University and were carried out in accordance with the Animal Experiment Guidelines of Wenzhou Medical University.

### 2.5. EPC Clone Formation Experiment

In order to evaluate the EPC colony forming unit (EPC-CFU), 1 × 10^6^ peripheral blood mononuclear cells of each group of mice were cultured in methylcellulose-containing medium M3236 (StemCell Technologies). Stem cell-derived factors are 20 ng/mL, 50 ng/mL vascular endothelial growth factor, 20 ng/mL IL-3, 50 ng/mL basic fibroblast growth factor, 50 ng/mL epidermal growth factor, 50 ng/mL insulin-like growth factor-1 (all from R&D Systems), 2 U/mL heparin (Sigma-Aldrich), and 10% FBS (Gibco), which were added. After culturing for 10–12 days, the EPC-CFU culture was treated with 0.4 mg/mL DiI-LDL (Biomedical Technologies) for 2 hours and fixed by applying 1 mL of 2% paraformaldehyde (PFA, Sigma-Aldrich) for 1 hour at room temperature. After washing the methylcellulose-containing medium with PBS, the culture was reacted with FITCBS-lectin 1 (Vector Laboratories) at room temperature for 1 hour. After washing with PBS, the culture was observed under a fluorescence microscope (IX70; Olympus). The number of EPC-CFU reflects the number of original EPCs in the initial classified cell fraction.

### 2.6. Establishment of the Lower Limb Ischemia Model

We established 30 male C57BL/6N mice critical limb ischemia models by ligating the femoral artery. The mice were divided into control group and model group. The mice in the control group did not do any treatment, and the mice in the model group were intraperitoneally anesthetized with midazolam (5 mg/kg) and medetomidine (0.5 mg/kg). The femoral artery was ligated and removed at the level of the inguinal ligament and knee joint. Seven days later, the blood supply rate of the mice was evaluated by laser Doppler imaging (LDI), and 10% of the mice whose blood flow on the affected side returned to 20% of the blood flow on the healthy side were defined as a critical limb ischemia model.

RETRACTED

### 2.7. Animal Grouping and Administration

The model mice were divided into (1) PBS group, (2) Cl-amidine group, and (3) AMD3100 group, 10 mice in each group. Peripheral blood mononuclear cells induced by Cl-amidine were injected intramuscularly into mice with lower limb ischemia. At the same time, peripheral blood mononuclear cells induced by PBS and AMD3100 were used as negative and positive controls to be injected into mice corresponding to lower limb ischemia. After 28 days, laser Doppler imager was used to observe the recovery of blood perfusion. After the test was completed, the mice were fasted for 12 hours, and peripheral blood was collected at the same time point, and then the mice were sacrificed to collect the ischemic gastrocnemius muscle. Nikon inverted fluorescence microscope was used to take pictures to observe the distribution and number of GFP-positive cells (endothelial cells) and to evaluate the number of EPCs by the number of green fluorescent protein; TUNEL staining method was used to observe cell apoptosis in ischemic tissues. Using immunofluorescence staining, BS-lectin 1 and anti-mouse CD31 antibody were used to identify endothelial cells in frozen tissue sections and observe the density of capillary formation.

### 2.8. Separation and Detection of EPCs

The peripheral blood of each group of mice was separated into EPCs according to the method described in Section 2.2, and MTT, Transwell, and related kits were used to detect cell proliferation, migration, and tubule formation ability.

Proliferation of EPCs: the cells cultured to the 7th day in each group were collected and counted. The same amount of EPCs was inoculated on a 96-well plate, and each group had 5 replicate wells. After the cells adhered, 20 *μ*L of 5% MTT was added, the supernatant was discarded after continuous incubation for 4 hours, and 150 *μ*L of dimethyl sulfoxide was added. Use 490 nm to measure the absorbance value in the microplate reader.

Migration of EPCs: the same amount of cell fluid collected from each group was added to the upper chamber of the Transwell chamber. The lower chamber was a culture medium containing 50 mg/L VEGF. After 1 day, it was rinsed with PBS, and 1 mL 4% paraformaldehyde was added to the lower chamber for fixation. 30 min after proper drying, we used Giemsa staining for 30 min, rinsed with PBS, and took out the filter cover, and 5 fields of view were randomly selected for counting.

RETRACTED

EPCs' ability to form small tubes: according to the kit operation, the Matrigel and the diluent were frozen and thawed overnight, and 100 *μ*L of the diluent was added to the 900 *μ*L of the glue and added to a 96-well plate, 50 *μ*L per well, incubated for 1 h to coagulate into gel. Cells of each group were seeded on the gel at 5 × 10^3^ EPCs/well; after 1 day of culture, the formation of tubules was observed under a microscope, and 5 fields of view were randomly selected for counting.

### 2.9. Statistical Method

All data were processed with SPSS 21.0 statistical software, and GraghPad Prism 8 was used to make statistical graphs. Measurement data are expressed as mean ± standard deviation ($\bar{x}$ ± *s*), independent sample *t*-test is used for comparison between groups, single-factor analysis of variance should be used for comparison between multiple groups, and Tukey's post hoc test is performed. *P* < 0.05 indicates that the difference is statistically significant.

## 3. Results

### 3.1. Expression of PAD4 in Peripheral Blood EPCs and Its Localization in Peripheral Arterial Disease

The results of the Dil-Ac-LDL uptake experiment showed that the uptake of Dil-Ac-LDL by EPCs isolated in peripheral blood showed red fluorescence, and the result was positive, indicating that the isolated cells were indeed functional EPCs, as shown in Figure 1(a). Q-PCR results showed that PAD4 was highly expressed in peripheral blood EPCs of peripheral artery disease, and the difference was statistically significant (*P* < 0.05), as shown in Figure 1(b). The immunofluorescence results showed that the overexpressed PAD4 accumulated in the nucleus after GSK3*β* incubation, as shown in Figure 1(c).

### 3.2. Influence of PAD4 on the Number and Function of EPCs

The results of the EPCs clone formation experiment showed that, compared with the PBS group, the Cl-amidine group and the AMD3100 group mouse peripheral blood mononuclear cell cultures detected more EPC-CFU, and the Cl-amidine group was more than the AMD3100 group, and the difference was statistically significant (*P* < 0.05), as shown in Figure 2(a). The cells glow red after ingesting Dil-ac-LDL, and the cells glow green when combined with FITC-UEA-1. The cells are differentiated EPCs after ingesting Dil-Ac-LDL and FITC-UEA-1 at the same time. The results show that The EPCs in the Cl-amidine group had the largest uptake activity, as shown in Figure 2(b).

RETRACTED

### 3.3. Effect of PAD4 on Blood Perfusion in Mice with Peripheral Arterial Disease

The results of blood perfusion showed that the blood perfusion index of mice in the model group was significantly lower than that in the control group, and the difference was statistically significant (*P* < 0.05), as shown in Figure 3(a). Compared with the PBS group, the blood perfusion index of the Cl-amidine group and the ADM3100 group was higher, and the Cl-amidine group was higher than that of the ADM3100 group. The difference was statistically significant (*P* < 0.05), as shown in Figure 3(b).

### 3.4. Effect of PAD4 on the Number of EPCs in Mice with Peripheral Arterial Disease

Observed under a fluorescence microscope, the gastrocnemius muscle tissue of the Cl-amidine group and the ADM3100 group formed more GFP and capillary blood vessels than the PBS group, and the apoptosis was less than that of the PBS group. The Cl-amidine group changed significantly compared with the ADM3100 group, and the difference was statistically significant (*P* < 0.05), as shown in Figures 4(a)–4(c).

### 3.5. Effect of PAD4 on the Function of EPCs in Mice with Peripheral Arterial Disease

The results of MTT and Transwell showed that, compared with the PBS group, the proliferation and migration ability of EPCs in the Cl-amidine group and the ADM3100 group was significantly enhanced, and the Cl-amidine group was stronger than the ADM3100 group, and the difference was statistically significant (*P* < 0.05), as shown in Figures 5(a) and 5(b).

### 3.6. Effect of PAD4 on the Formation of Capillaries in Mice with Peripheral Arterial Disease

The results of the angiogenesis experiment showed that, compared with the PBS group, the formation of tubules in the Cl-amidine group and the ADM3100 group was significantly increased, and the Cl-amidine group was more than the ADM3100 group, and the difference was statistically significant (*P* < 0.05), as shown in Figure 6.

## 4. Discussion

Arteries help transport blood rich in oxygen and various nutrients to various parts of the body. When the arteries of the lower extremities are blocked, they cannot get enough blood or oxygen, causing arterial ischemia. At this time, it is called peripheral arterial disease. Peripheral arterial disease is a fatal systemic disease, caused by atherosclerosis, which can cause cardiovascular and cerebrovascular diseases to increase by 2 to 6 times [10]. According to reports [11, 12], the overall prevalence of peripheral arterial disease in adults is 12%. Risk factors include advanced age, young men, smoking, diabetes, hypertension, and dyslipidemia, which are characterized by coronary arteries and cerebrovascular diseases. The risk of events increases, with carotid artery stenosis rates ranging from 15% to 25% and coronary artery disease rates from 30% to 50%. Because peripheral arterial disease has a greater impact on body functions, finding and exploring a treatment plan that can reduce the symptoms of peripheral arterial disease and avoid amputation without affecting the normal walking function of the body is an ideal goal for the treatment of patients with peripheral arterial disease.

RETRACTED

Although a variety of treatment methods have been proposed one after another, these methods mainly include drug therapy (including antiplatelet therapy), exercise therapy, and revascularization surgery. Among these methods, revascularization surgery has surgical risks (mainly the risks of intravascular manipulation), and it is not recommended to use it if there is no ischemia that endangers the limbs. Therefore, under normal circumstances, patients with peripheral arterial disease will be recommended to use conservative medication and exercise therapy [13]. In terms of drug treatment, cilostazol was recognized as the first-line drug for the treatment of peripheral artery disease in the clinical guidelines issued by the American College of Cardiology and the American Heart Association in 2005 [14]. However, the use of cilostazol can also produce certain side effects, which mainly include dizziness and diarrhea. The most serious is that it may cause a certain burden on the cardiovascular system and lead to heart failure. Therefore, exploring safer and more effective treatment methods has become a hot spot in the study of peripheral arterial disease.

Studies have found that endothelial progenitor cells have the ability to enhance neovascularization in the case of ischemia and can exert a therapeutic effect around blocked blood vessels that require reperfusion. In addition, the results of animal experiments confirmed that EPCs derived from peripheral blood or bone marrow have the function of promoting angiogenesis and accelerating the recovery of blood supply in ischemic tissues [15–17]. In addition, recent studies have shown that endothelial progenitor cells in peripheral blood also have the function of repairing damaged vascular endothelium, so they can be used as a reservoir for endothelial cells [18]. However, EPCs mainly exist in the bone marrow, and the content in peripheral blood is very small. Peripheral blood EPCs only account for 0.01% of peripheral cells. However, when the body has ischemia, vascular injury, or burns or is under the action of exogenous cytokines, EPCs will change; they are mobilized from bone marrow to peripheral blood and then enter the systemic circulation to reach the injured site, thereby promoting endothelial repair and neovascularization [19, 20]. Animal experiments have confirmed that the degree of local tissue ischemia is related to the number of EPCs in peripheral blood [21]. Therefore, we speculate that increasing the number of EPCs will help repair the ischemic tissue and treat peripheral arterial disease. Studies have shown that inhibiting PAD can reduce the burden of atherosclerosis and the formation of arterial thrombosis by blocking the extracellular trapping network of neutrophils and regulating the innate immune response. It is clear that PAD can participate in the treatment of cardiovascular-related diseases. PAD4 can also regulate hematopoietic stem cells that share the same origin with EPCs. Therefore, we put forward a conjecture whether PAD can play a role in peripheral arterial disease by regulating EPCs.

RETRACTED

In order to confirm this conjecture, we collected peripheral blood from patients with peripheral artery disease and separated EPCs for identification and testing. The results showed that EPCs can successfully take up Dil-Ac-LDL, and the uptake capacity of Dil-Ac-LDL is the functional capacity of the endothelial cell lineage, confirming the successful isolation of EPCs. Q-PCR detection revealed that PAD4 was highly expressed in peripheral blood EPCs of peripheral arterial disease and accumulated in the nucleus. It is suggested that the high expression of PAD4 may be involved in the pathological response of peripheral arterial disease. Studies have confirmed that AMD3100, a small molecule chemical antagonist of CXCR4, can quickly and effectively mobilize endothelial progenitor cells and circulating angiogenic cells to achieve the effect of treating lower limb ischemia [22]. In order to explore whether PAD4 can regulate EPCs, in the subsequent experiments, PBS was used as a negative control and AMD3100 was used as a positive control. We injected mice with PAD4 inhibitor Cl-amidine and collected peripheral blood mononuclear cells for EPCs clone formation experiments. The results showed that more EPC-CFU was detected in the peripheral blood mononuclear cell cultures of mice injected with Cl-amidine, and the activity of both uptake of Dil-Ac-LDL and binding to FITC-UEA-1 was the strongest, indicating that Cl-amidine can increase the number of EPCs and enhance its uptake function.

In order to explore the regulatory and therapeutic effects of PAD4 on EPCs in peripheral arterial disease, we established a mouse lower limb ischemia model as a peripheral arterial disease model. The blood perfusion experiment showed that the blood perfusion index of the model group was significantly lower than that of the control group, suggesting that the peripheral arterial disease and model mice were successfully established. The blood perfusion index of mice injected with Cl-amidine and ADM3100 mononuclear cells was higher than that of mice injected with PBS mononuclear cells, and the Cl-amidine group was higher than the ADM3100 group. It shows that inhibiting PAD4 has a certain effect on improving the blood flow recovery of peripheral arterial disease. The study also found that PAD4 inhibitors can increase EPCs and blood vessel formation in the gastrocnemius muscle tissue of mice with peripheral artery disease and reduce cell apoptosis. The function of EPCs in PAD4 mice with peripheral arterial disease was observed. Compared with the PBS group, the proliferation, migration, and tubule formation ability of EPCs in the Cl-amidine group and the ADM3100 group were significantly enhanced, and the Cl-amidine group was stronger than the ADM3100 group. It is suggested that the inhibition of PAD4 can increase the number of EPCs in peripheral arterial disease and can enhance their proliferation, migration, and tubule function, thereby achieving disease amelioration, which confirms the above conjecture.

RETRACTED

In summary, PAD4 is highly expressed in peripheral arterial diseases. The PAD4 inhibitor Cl-amidine can increase the number of EPCs and can treat peripheral arterial diseases by improving the proliferation, migration, and vascularization of EPCs. This study helps us understand the changes of EPCs in peripheral arterial disease and the influence of PAD4 on the function of EPCs and provides data support for the exploration of the pathogenic mechanism of peripheral vascular disease and the formulation of corresponding treatment measures.

## Figures and Tables

**Figure 1:** The expression of PAD4 in peripheral blood EPCs and its localization in peripheral arterial disease (200x). (a) Dil-Ac-LDL fluorescence detection to identify EPCs; (b) Q-PCR detection of PAD4 expression in peripheral blood EPCs of peripheral arterial disease; (c) immunofluorescence detection of PAD4 location in cells; compared with healthy people, ^*∗*^*P* < 0.05.

**Figure 2:** The influence of PAD4 on the number and function of EPCs (200x). (a) EPCs clone formation experiment to detect the number of EPC-CFU; (b) Dil-Ac-LDL and FITC-UEA-1 fluorescence detection of EPCs function; compared with the PBS group, ^*∗*^*P* < 0.05; compared with ADM3100 group, ^#^*P* < 0.05.

**Figure 3:** The effect of PAD4 on blood perfusion in mice with peripheral arterial disease. (a) The blood perfusion of mice in the control group and the experimental group; compared with the control group, ^*∗*^*P* < 0.05; (b) the blood perfusion of the three groups of mice; compared with the PBS group, ^*∗*^*P* < 0.05; compared with the ADM3100 group, ^#^*P* < 0.05.

RETRACTED

**Figure 4:** The effect of PAD4 on the number of EPCs in mice with peripheral artery disease (200x). (a) Nikon inverted fluorescence microscope to observe the distribution and number of GFP-positive cells (EPCs); (b) TUNEL staining method to observe cell apoptosis in ischemic tissue; (c) immunofluorescence staining, using BS-lectin 1 and anti-mouse CD31 antibody, showing the density of capillary formation; compared with the PBS group, ^*∗*^*P* < 0.05; compared with the ADM3100 group, ^#^*P* < 0.05.

**Figure 5:** The effect of PAD4 on the function of EPCs in mice with peripheral artery disease (200x). (a) MTT detects the proliferation ability of EPCs; (b) Transwell detects the migration ability of EPCs; compared with the PBS group, ^*∗*^*P* < 0.05; compared with the ADM3100 group, ^#^*P* < 0.05.

**Figure 6:** The effect of PAD4 on capillary formation in mice with peripheral artery disease (200x). The angiogenesis experiment observes tubule formation; compared with the PBS group, ^*∗*^*P* < 0.05; compared with the ADM3100 group, ^#^*P* < 0.05.

## Data Availability

The datasets used and/or analyzed during the current study are available from the corresponding author on reasonable request.
